# Deep Learning of Subject Context in Ideological and Political Class Based on Recursive Neural Network

This article has been retracted.

**DOI:** 10.1155/2022/8437548

**Published:** 2022-09-30

**Authors:** Tingting Jiang, Xiang Gao

**Affiliations:** ^1^School of Marxism, Guangxi University of Chinese Medicine, Nanning 530200, China; ^2^School of Public Health and Management, Guangxi University of Chinese Medicine, Nanning 530200, China

## Abstract

Ideological and political education is the most important way to cultivate students' humanistic qualities, which can directly determine the development of other qualities. However, at present, the direction of ideological and political innovation in higher vocational colleges is vague. In response to this problem, this study proposes a model based on HS-EEMD-RNN. First, the ensemble empirical mode decomposition (EEMD) method is used to decompose the measured values, and then the recurrent neural network (RNN) is used to train each component and the remaining items. Finally, through the mapping relationship obtained by the model, the response prediction value of each component and the remaining items can be obtained. In the RNN training process, the harmony search (HS) algorithm is introduced to optimize it, and the noise is systematically denoised. Perturbation is used to obtain the optimal solution, thereby optimizing the weight and threshold of the RNN and improving the robustness of the model. The study found that, compared with EEMD-RNN, HS-EEMD-RNN has a better effect, because HS can effectively improve the training and fitting accuracy. The fitting accuracy of the HS-EEMD-RNN model after HS optimization is 0.9918. From this conclusion, the fitting accuracy of the HS-EEMD-RNN model is significantly higher than that of the EEMD-RNN model. In addition, four factors, career development, curriculum construction, community activities, and government support, have obvious influences on ideological and political classrooms in technical colleges. The use of recurrent neural networks in the research direction of deep and innovative research on the subject context of ideological and political classrooms can significantly improve the prediction accuracy of its development direction.

## 1. Introduction

At present, the most fundamental task is to improve the overall quality of students, which is also the goal of social development. To cultivate socialist successors, schools, society, and families must cooperate closely to carry out student education from the basics and improve students' comprehensive quality. In education, ideological and political courses can play an extremely important role. Therefore, colleges and universities should take responsibility and regard cultivating students' correct thinking as one of the most important educational tasks [1]. The education of ideological and political courses is the most important way to cultivate students' humanistic qualities. Ideological and political education is the most important way to cultivate students' humanistic qualities. Quality in the broad sense mainly refers to material and spirit and is a quality both inside and outside, which contains extremely rich contents and can be divided into political and other aspects of quality [2]. Ideological quality plays a decisive role, so the most fundamental goal of school education is to cultivate talents with all-around development of morality, intelligence, physique, aesthetics, and labor and must have certain consciousness and scientific and technological knowledge. Ideological and political quality can directly determine the development of other qualities. No matter what kind of career students will engage in in the future, they must establish the correct three views. Only students with good ideology and morality can guide the correct development of other qualities and provide a steady stream of spiritual power [3]. Therefore, innovative research in the ideological and political classroom is indispensable.

Foreign countries have civic education to carry out ideological domination of citizens and the corresponding expression of civic education discourse [4]. After the twentieth century, ideological and political education gradually formed two schools of universities based on historical research, namely, structuralism and functionalism [5]. Saussure founded thestructuralism school of ideological and political thinking, definingideological and political thinking as a science based on symbols and meanings.They advocated the study of the framework outline, practical operation, andsignificance of ideological and political thinking in daily life[6]. The functionalist ideological and political school advocates that more attention should be paid to the connotation of language itself, rather than to the external form and logical structure of ideological and political thinking. The ideological and political system can choose semantics independently, and the connotation of language is also transmitted [7]. Since the middle of the twentieth century, western discourse studies have gradually expanded from ideological and political studies to several related disciplines, such as philosophy, sociology, history, and literature. For example, Wittgenstein, a British philosopher, studied the relationship between ideology and politics and the external world, while Derrida, a French philosopher, believed that, to understand the specific practice of society, it is necessary to analyze ideology and politics [8]. After the 1960s, preliminary discussions on ideological and political studies began to appear in the field of sociology [9]. By comparing the studies of sociology by famous scholars, we can see their efforts in ideological and political studies, such as those of Habermas and Foucault. Habermas elaborated on the four principles of ideological and political discourse, which laid a foundation for the development of ideological and political studies. Foucault believed that discourse “covers various forms of formal or informal verbal interaction and written texts.” “Discourse is power, and people give themselves to power through discourse” [10]. To solve the problem of the nonstationarity of signals, Huang et al. [11] proposed the empirical mode decomposition (EMD) method in 1998. However, the signal envelope of this algorithm is prone to shape distortion and causes an endpoint effect, which makes the decomposition of each component inaccurate. Some researchers [12] proposed EEMD, which can effectively solve the shortcomings of the above EMD algorithm. EEMD algorithm has been widely used. For example, some researchers used EEMD-RBF neural network to build a model of ideological and political direction [13]. Some scholars realized the extraction of key factors of ideological and political education through the EEMD algorithm [14]. Based on EEMD-JADE, some researchers have better isolated the environmental factors [15]. To improve training fitting and prediction accuracy, the recurrent neural networks (RNN) algorithm is introduced. RNN is a kind of structure-optimized neural network, which introduces a cyclic structure in the hidden layer and carries out internal connections among the hidden elements. During training, information can be propagated forward or backward in the model, which can improve the training efficiency and accuracy. At present, there are a lot of research achievements on the application of this algorithm. For example, researchers predicted the thematic context of ideological and political education through RNN and its fusion method [16]. Some researchers constructed a combination algorithm of CNN and RNN to explore continuous identity authentication in free text keystroke mode [17]. Some researchers also studied the necessity [18]. In the subject innovation of ideological and political class, the predicted value contains the prediction error and system noise, in order to further improve the precision of training fitting and the robustness of the algorithm.

In conclusion, it is difficult for a single algorithm model to solve complex problems, while, for the innovation of ideological and political classroom in higher vocational colleges affected by complex conditions, which is random and nonlinear, it is more difficult to achieve high precision prediction [19, 20]. Therefore, to overcome the shortcomings of the single algorithm, such as easily falling into the local minimum of the error function, slow convergence speed, and excessive convergence, this paper first uses the EEMD algorithm to smooth the displacement data. Then, using the strong nonlinear mapping ability of the RNN neural network, the harmony search algorithm was used to denoise and optimize it, and the advantages of each algorithm were integrated to improve the displacement prediction accuracy and model calculation efficiency, and the HS-EEMD-RNN ideological and political classroom prediction model was constructed. Recurrent neural networks have significantly improved the prediction accuracy of innovative directions in ideological and political classrooms and improved the use of computer network algorithms for practical applications and other such research.

## 2. Principles and Methods

### 2.1. Ensemble Empirical Mode Decomposition (EEMD)

The EEMD algorithm adds enough normal distributed white noise into the original time series [21] and meanwhile performs EMD decomposition on the new time series. Then, the arithmetic average of each decomposition quantity is taking advantage of the property that the mean value of white noise is zero, and the IMF component and the remaining term R of EEMD decomposition can be obtained [22]. The decomposition steps are as follows:

(1) Considering that there are some problems in ideological and political prediction, the prediction is not accurate. In this study, we first add equal-length Gaussian white noise *N* times to the original time series to obtain several new time series:
  (1) $$\begin{array}{c} y_{i}\left(t\right)=y\left(t\right)+n_{i}\left(t\right)\text{,} \end{array}$$
where *y*_*i*_(*t*) is the time series after adding white noise for the *i*-th time, *y*(*t*) is the original time series, and *n*_*i*_(*t*) is normally distributed white noise signal.
(2) Then, the EMD algorithm is used to decompose the new time series with white noise, and the eigenmodal function and a residual term can be obtained:
  (2) $$\begin{array}{c} y_{i}\left(t\right)=\overset{J}{\underset{i=1}{\sum }}w_{ij}\left(t\right)+r_{i}\left(t\right)\text{,} \end{array}$$
where *w*_*ij*_(*t*) is the *j*-th eigenmode function component obtained after adding white noise for the *i*-th time and *r*_*i*_(*t*) is the residual term.
(3) Then *N* groups of intrinsic components and residual term *r*(*t*) are averaged to obtain the final *IMF* component and residual quantity *R*(*t*).
  (3) $$\begin{array}{c} y_{i}\left(t\right)=\overset{J}{\underset{i=1}{\sum }}w_{ij}\left(t\right)+r_{i}\left(t\right)\text{,}\\ R\left(t\right)=\frac{1}{N}\overset{N}{\underset{i=1}{\sum }}r_{i}\left(t\right)\text{,} \end{array}$$
where *IMF*_*j*_(*t*) denotes the final decomposition component of EEMD and *R*(*t*) is the final surplus.
(4) Finally, the original time series signal can be decomposed into
  (4) $$\begin{array}{c} y\left(t\right)=\overset{J}{\underset{j=1}{\sum }}IMF_{j}\left(t\right)+R\left(t\right)\text{.} \end{array}$$

### 2.2. RNN Model

 The advantage of RNN lies in the one-time activation of different neuralunits, that is, the output content of hidden layer nodes at the previous timecan not only reflect the time, but also be used as the input of the next outputlayer. At the same time, after processing the information at this moment, itcan lead to the hidden layer node at the next time point [23]. Compared with traditional neural networks, RNN can improve the convergence speed and training accuracy in the process of training fitting and predicting displacement [23].

RNN is a recursive process in the time dimension. The results of the previous time have a direct impact on the training for the next time. However, because the weights at each time step are the same, different units at the same time will share the same group weights [24]. For a sequence *x* of length *T*, the size of the input layer of the RNN is *I*, the size of the hidden layer is *H*, the size of the output layer is *K*, and the dimensions of the three weight matrices *U*, *V*, and *W* can be obtained:

(5) $$\begin{array}{c} \left\{\begin{array}{c} U\in R^{l\times H}\\ W\in R^{H\times H}\text{,}\\ V\in R^{H\times K} \end{array}\right. \end{array}$$

where *x*^*t*^ is the input of the *t*-th neuron in the sequence, *a*^*t*^ is the input of the *t*-th hidden layer, and *b*^*t*^ is the nonlinear activation of *a*^*t*^, that is, the output of the neural network. Therefore, *a*^*t*^ is determined by the input layer and the output *b*^*t*−1^neuron of the previously hidden layer:

(6) $$\begin{array}{c} a_{h}^{t}=\underset{i}{\sum }w_{ih}x_{i}^{t}+\underset{h^{\prime }}{\sum }w_{h^{\prime }h}b_{h^{\prime }}^{t-1}\text{,}\\ b_{h}^{t}=f\left(a_{h}^{t}\right)\text{.} \end{array}$$

The innovation sequence of the ideological and political classroom starts from *t* = 1, so *b*_0_ = 0, and then the information of the hidden layer is transmitted to the output layer, and the output result of the output layer is

(7) $$\begin{array}{c} a_{k}^{t}=\underset{h}{\sum }w_{hk}b_{h,}^{t}\\ y_{k}^{t}=\frac{e^{a_{k}^{t}}}{\underset{j}{\sum }e^{a_{j}^{t}}}\text{.} \end{array}$$

At time *t*, the residual of the ordinary neural network is *δ*_*k*_^*t*^ = *y*_*k*_^*t*^ − *z*_*k*_^*t*^, Since the hidden layer of RNN needs to accept the signal of the hiddenlayer at the previous time in forward conduction and the feedback of the hiddenlayer at the next time in reverse conduction, the residual term of RNN outputlayer is as follows:

(8) $$\begin{array}{c} \delta_{h}^{t}=f^{\prime }\left(a_{h}^{t}\right)\left(\underset{k}{\sum }\delta_{k}^{t}w_{hk}+\underset{h^{\prime }}{\sum }\delta_{h^{\prime }}^{t+1}w_{hh^{\prime }}\right)\text{.} \end{array}$$

When the length of the displacement sequence is *T*, the residual *δ*^*T*+1^ is all 0, and the entire network has only one set of parameters *U*, *V*, and *W*, then the reciprocal of time *t*:

(9) $$\begin{array}{c} U:\frac{\partial O}{\partial w_{ih}}=\frac{\partial O}{\partial a_{h}^{t}}\frac{\partial a_{h}^{t}}{\partial w_{ih}}=\delta_{h}^{t}x_{i}^{t}\text{,}\\ V:\frac{\partial O}{\partial w_{hk}}=\frac{\partial O}{\partial a_{k}^{t}}\frac{\partial a_{k}^{t}}{\partial w_{hk}}=\delta_{k}^{t}b_{h}^{t}\text{,}\\ W:\frac{\partial \theta }{\partial w_{h^{\prime }h}}=\frac{\partial \theta }{\partial a_{h}^{t}}\frac{\partial a_{h}^{t}}{\partial w_{h^{\prime }h}}=\delta_{k}^{t}b_{h^{\prime .}}^{t}. \end{array}$$

Then it can be written in the unified form (assuming *x*_*i*_^*t*^ = *a*_*i*_^*t*^ = *b*_*i*_^*t*^ for the input layer):

(10) $$\begin{array}{c} \frac{\partial O}{\partial w_{hij}}=\frac{\partial O}{\partial a_{h}^{t}}\frac{\partial a_{j}^{t}}{\partial w_{ij}}=\delta_{j}^{t}b_{i}^{t}\text{.} \end{array}$$

Finally, for time *t* = 1, 2,…, *T*, by summing the recursion of the RNN neural network, the derivative of the RNN network concerning the weight parameter can be obtained:

(11) $$\begin{array}{c} \frac{\partial O}{\partial w_{ij}}=\frac{\partial O}{\partial a_{h}^{t}}\frac{\partial a_{j}^{t}}{\partial w_{ij}}=\underset{t}{\sum }\delta_{j}^{t}b_{i}^{t}\text{.} \end{array}$$

### 2.3. Harmony Search Algorithm

For the displacement components obtained by EEMD decomposition, the high-frequency components are mainly caused by monitoring error noise, especially the IMF_1_ component, so it is necessary to systematically denoise them [25]. The basic idea of the harmony search algorithm is a metaheuristic optimization algorithm that imitates the harmony tuning process played by a band. The implementation process of optimizing the RNN neural network is as follows [26]:

Step 1: Initialize the relevant algorithm parameters.
HMS determines the global search capability of the HS algorithm, but an excessively large HMS value will affect the speed of convergence to the optimal solution. A large HMCR value is beneficial to the local search of the algorithm. The specific values of algorithm parameters can be determined by simulation experiments [27].
Step 2: Define the objective function and initialize the harmony memory.
Define the objective function: the average relative error *F* between the expected output (measured value) and the network output (fitted value), where the smaller the *F* value, the better the degree of optimization.
  (12) $$\begin{array}{c} F=\frac{1}{H}\overset{H}{\underset{i=1}{\sum }}\frac{\left|y^{\prime }\left(i\right)-y\left(i\right)\right|}{\left|y\left(i\right)\right|}\text{,} \end{array}$$
where *H* is the total number; *y*′(*i*) and y(*i*) are the measured and fitted values of the *i*-th sample, respectively.
Construct *HMS* random initial harmonics *x*^1^, *x*^2^,…, *x*^*HMS*^ to add a harmonic memory bank and the harmony *x*_*i*_ in the memory; the bank corresponds to a set of weights and thresholds of the RNN neural network. The harmony memory bank is
  (13) $$\begin{array}{c} HM=\left[\begin{array}{cc} x^{1} & f\left(x^{1}\right)\\ x^{2} & f\left(x^{2}\right)\\ \vdots & \vdots \\ x^{HMS} & f\left(x^{HMS}\right) \end{array}\right]=\left[\begin{array}{ccccc} x_{1}^{1} & x_{2}^{1} & \cdots & x_{N}^{1} & f\left(x^{1}\right)\\ x_{1}^{2} & x_{2}^{2} & \cdots & x_{N}^{2} & f\left(x^{2}\right)\\ \vdots & \vdots & \ddots & \vdots & \vdots \\ x_{1}^{HMS} & x_{N}^{HMS} & \cdots & x_{N}^{HMS} & f\left(x^{HMS}\right) \end{array}\right]\text{,} \end{array}$$
where *x*_*j*_^*i*^ is the *j*-th weight or threshold of the *i*-th group of harmony in the RNN network and *f*(*x*^*i*^) denotes the *i*-th group of objective function values, that is, the average relative error between the *i*-th group of network outputs and the expected output.
Step 3: Create new harmonies.
To create new harmony is to construct new solution vectors. According to the harmony learning memory bank, tune tuning, randomly generate the tone *y*′(*j* = 1, 2,…, *N*) of the new harmony:
  (14) $$\begin{array}{c} x_{j}^{\prime }=\left\{\begin{array}{cc} x_{j}^{\prime }\in \left(x_{j}^{1},x_{j}^{2},\cdots ,x_{j}^{HMS}\right) & r_{1}<HMCR\\ x^{L}+r_{1}\left(x^{U}-X^{L}\right) & r_{1}⩾HMCR \end{array}\right.\text{,} \end{array}$$
where *r*_1_ represents random value within [0, 1]. *x*_*j*_′*ϵ*(*x*_*j*_^1^, *x*_*j*_^2^,…, *x*_*j*_^*HMS*^) is the randomly selected component in the *j*-th column HMS; *Z* represents the upper and lower limits of the JTH column. *x*^*U*^ and *x*^*L*^ are the upper and lower limits of the value of the *j*-th column components. Equation (14) shows that, for any new tone, it will be selected from the memory library with the probability of HMCR, and the value will be randomly selected from its corresponding value interval with the probability of 1-HMCR [23]. If *x*_*j*_′ is the solution component in the harmony memory, it is fine-tuned as
  (15) $$\begin{array}{c} x_{j}^{\prime }=\left\{\begin{array}{cc} x_{j}^{\prime }+r_{3}bw & r_{2}<PAR\\ x_{j}^{\prime } & r_{2}⩾PAR \end{array}\right.\text{,} \end{array}$$
where *r*_1_ and *r*_2_ are distributed random values in [0, 1] and [−1, 1], respectively.
Step 4: Update the memory bank.
Step 5: End the loop.

Repeat steps 3 and 4 until the termination criterion is met or the maximum number of iterations is reached.

### 2.4. Modeling Process

Based on the advantages of the above algorithms, the specific modeling process of the EEMD-RNN combination model based on HS optimization is as follows:

1. Determine the research measurement points of the influencing factors of the ideological and political classroom theme, decompose the measurement values through EEMD, and obtain several groups of IMF components and residual items R.
2. The RNN neural network algorithm is used to train and fit the IMF component and the residual item R. The input is the environmental quantity and the time-dependent variable, and the output is the key influencing factor. During the training process, the thresholds and weights of the RNN are optimized through the harmony search (HS) algorithm until the optimal solution is obtained.
3. Calculate the IMF component and residual item R corresponding to the prediction set by training the optimal fitting mapping relationship.
4. Equal weight summation of the predicted values of each component displacement IMF and the remaining term R is the final prediction result.

### 2.5. Model Accuracy Assessment

To evaluate prediction accuracy, MAE, RMSE, and MAPE are applied to evaluate the accuracy [28], which are expressed as

(16) $$\begin{array}{c} MAE=\frac{1}{n}\overset{n}{\underset{t=1}{\sum }}\left|Y_{t}-{\hat{Y}}_{t}\right|\text{,}\\ RMSE=\sqrt{\frac{1}{n}\overset{n}{\underset{t=1}{\sum }}{\left(Y_{t}-{\hat{Y}}_{t}\right)}^{2},}\\ MAPE=\frac{1}{n}\overset{n}{\underset{t=1}{\sum }}\left|\frac{Y_{t}-{\hat{Y}}_{t}}{Y_{t}}\right|\text{,} \end{array}$$

where *Y*_*t*_ is the measured value of the influencing factors of the ideological and political classroom, $\hat{Y_{t}}$ is the calculation amount of the model, *n* is the total amount of monitoring data, and *t* is the time corresponding to the monitoring data.

## 3. Experimental Procedure and Result Analysis

### 3.1. Data and Factor Selection

The scientific advancement of ideological and political course teaching activities in technical colleges requires the improvement of course design as support. It is necessary to focus on teaching design and actively explore the construction of a scientific teaching planning system to ensure that ideological and political courses can be displayed to the greatest extent. The advantages of teaching design have significantly improved the quality of talent training in technical schools. This study mainly selects relevant classrooms and students and teachers as the research objects, selects the experimental samples as the actual values of the experiment, and selects the influencing factors as career development, curriculum construction, community activities, government support, family education, teacher-student environment, and other factors. Seven schools in a city were selected as the experimental data source.

### 3.2. Test Analysis

There are two EEMD decomposition parameters: the standard deviation *Nstd* of white Gaussian noise is generally 0.01∼0.4, and the number of noise additions NE is generally 50 or 100. To obtain the best decomposition result, the comprehensive *Nstd* is 0.01, and the NE is 100. The EEMD decomposition results of the training set of the model are shown in Figure 1, in which 7 groups of IMF components and 1 group of residual *R*, IMF_1_, IMF_2_, and IMF_3_ components are high-frequency components, and the remaining IMF components are low-frequency components. For high-frequency components, it is mainly caused by monitoring error noise, especially the IMF1 component. Therefore, systematic denoising is necessary to improve model accuracy.

To reduce the interference of noise errors in the measured values to the training results, in the process of optimizing the RNN training process of the harmony search algorithm, the size of the harmony memory bank *HMS* is 100, and the search range is [−1, 1]. The retention probability HMCR of the harmony memory is 0.85, the pitch fine-tuning probability PAR is 0.2, and the fine-tuning step size *bw* is 0.2. After the training of the HS optimized RNN, the fitting values of each component *IMF* and the residual R are equally weighted to obtain the fitting value of the displacement. The fitting result is shown in Figure 2.

At the same time, compared with the fitting results of the EEMD-RNN model, the fitting accuracy is demonstrated in Table 1. The EEMD-RNN model alone has a fitting accuracy of 0.9865, while the HS-EEMD-RNN model optimized by the HA algorithm has a fitting accuracy of 0.9918, and the fitting accuracy of the HS-EEMD-RNN is significantly higher.

The network trained by HS-EEMD-RNN is used to predict the displacement IMF of each component and the remaining term R, and the equal weight summation is the final dam displacement prediction result. At the same time, the displacement prediction value of EEMD-RNN is calculated, and the displacement prediction result is shown in Figure 3. Using MAE and RMSE as well as MAPE, three indicators are employed to evaluate the predictions of the two models, which are demonstrated in Table 2. The comparison results reveal that the HS-EEMD-RNN is better than the EEMD-RNN, which can meet the prediction requirements of the ideological and political classroom.

Among them, the sudden jump point in the change process is generally the focus of ideological and political classroom prediction, and the overfitting of the previous model and the large prediction error occurred more at the sudden jump point, so the EX5 displacement process line was selected to have the largest jump degree. The measured values of the seven factors are compared with the predicted values of the model to better evaluate the prediction accuracy of the model. It can be observed from Table 3 that the average absolute percentage error of HS-EEMD-RNN is 8.91%, which is significantly lower than 27.17% of EEMD-RNN.

The error analysis between the predicted values obtained from the proposed HS-EEMD-RNN model and the actual value predictions shows that four factors, career development, curriculum building, club activities, and government support, have a more significant impact on the civic science classroom in technical colleges. Therefore, innovations are made based on such factors, as shown in Section 3.3.

### 3.3. Innovation Direction Prediction Results

 In the basis of clear teaching design, to improve thecomprehensive effect of ideological and political course teaching activities intechnical schools, teachers should pay attention to choosing different entry points to reform and innovate theteaching mode and teaching a path and play therole of ideological and political teaching. In addition, students should begiven active guidance from multiple perspectives, so that they can activelyparticipate in the study and practice of ideological and political knowledge,so as to strengthen their professional quality and effectively ensure thatideological and political teaching activities achieve remarkable results.

1. Based on career development, strengthen professional ethics education
2. Good career development is a key concern of technical school students. In the process of carrying out ideological and political education forstudents, teachers should take students' professional growth and careerdevelopment as the basis, effectively carry out ideological and politicaleducation for students' vocational ability and ensure that students'professional ability and professional level are significantly improved. At thesame time, it is necessary to strengthen the professional ethics of students toensure that the teaching effect and the comprehensive quality of personneltraining work can be maximally promoted.
3. Build quality courses and guide students to explore
4. There is a close connection between the efficiency of technical schools and the innovation of curriculum in the process of implementing ideological education and guidance to students. Combined with the practical needs of talent training in technical schools, improve the construction of ideological and political courses to ensure that students can implement active and effective teaching guidance, so that the level of ideological awareness of students in technical schools can be continuously improved, and the training of talents in technical schools can be improved. Teachers of ideological and political courses in technical schools can systematically plan the needs of students' career development. Then, according to the personal growth needs and career development needs of students, explore the construction of basic curriculum systems such as employment and entrepreneurship guidance courses, legal basic knowledge courses, mental health education courses, current affairs, and politics courses, and create excellent ideological and political courses to improve education effect. At the same time, based on the construction of quality courses, the school should combine the application of information technology to build a platform, and political education can be provided from multiple perspectives. The development of class teaching activities provides rich talent support; effective guarantees are further optimized, as well as systematic advancement of talent training.
5. Carefully plan community activities and build an experience platform
6. In the practice of talent training in technical colleges, it is necessary not only to construct excellent courses from the perspective of theoretical education and guide students to systematically explore ideological and political content but also to consciously build experiential learning for students. The platform guides students to conduct a diversified exploration of the content of ideological and political courses. Positive educational guidance can be implemented for students. The goal becomes achieving all-around development and training students to become political education talents widely recognized by society.
7. Strengthen government support and build an ideological education platform
8. In the process of reforming and innovating, the leadership of schools and the support of enterprises are important, so that the students of technical colleges can enjoy themselves. Professional ability, moral cultivation, and so forth have been comprehensively improved to optimize the talent cultivation work of technical schools as a whole. The development of effective teaching activities needs to be supported by a sound policy system. Only local governments increase their support for technical schools and combine the needs of technical talents in the region to build a comprehensive and flexible system, adapt to the principles and policies of the talent development direction of technical schools, and further optimize the job training work and ideological and moral education work of technical school students to create a positive and healthy talent training environment in the educational practice of technical schools. Gradually improve and then optimize the overall efficiency of the construction of high-quality technical personnel in technical colleges.

## 4. Conclusion

To better determine the influencing factors of the theme of ideological and political classrooms, this paper uses environmental variables and time-sensitive variables as input, and the output is the key influencing factor, which is used to build the HS-EEMD-RNN model, so it can efficiently determine the research points of ideological and political classrooms. Through experimental analysis, the model based on HS-EEMD-RNN achieves better prediction accuracy than that based on EEMD-RNN. The experimental results show that some influencing factors selected in this paper, including career development, curriculum construction, community activities, government support, family education, and teacher-student environment, have played a key role in the ideological and political classroom. Good prediction accuracy can clarify teaching design and improve ideological and political classroom teaching activities in technical schools. At the same time, students can more actively participate in the learning and practice of ideological and political knowledge, strengthen their professional quality, and effectively ensure that ideological and political teaching activities can achieve significant results.

Based on the HS-EEMD-RNN model, this study analyzes the influencing factors of ideological and political education in higher vocational colleges and predicts the innovation direction of ideological and political classrooms. The study finds that HS-EEMD-RNN has better effects than EEMD-RNN, and the specific conclusions are as follows:

1. The HS can elevate and prove the training and fitting accuracy. The fitting accuracy of the EEMD-RNN model alone is 0.9865, while the fitting accuracy of the HS-EEMD-RNN model optimized by the HS algorithm is 0.9918. The fitting accuracy is significantly higher.
2. The average absolute percentage error of the HS-EEMD-RNN model is 8.91%, which is significantly lower than 27.17% of the EEMD-RNN model. The prediction accuracy of the HS-EEMD-RNN is better than that of the EEMD-RNN, meeting the forecasting requirements of ideological and political classrooms.
3. The influence of career development, curriculum construction, community activities, and government support on ideological and political classes in technical colleges is obvious; that is, the innovation direction should be based on career development, building excellent courses, elaborately planning community activities, and strengthening government support.

## Figures and Tables

**Figure 1:** EEMD decomposition results.

**Figure 2:** Fitting results between two models and actual values.

**Figure 3:** Comparison of prediction accuracy between EEMD-RNN model and HS-EEMD-RNN model.

**Table 1:** Comparison of fitting accuracy of the two models.

Models	R	MAE	RMSE	MAPE
EEMD-RNN	0.9865	0.197	0.207	0.107
HS-EEMD-RNN	0.9918	0.074	0.086	0.041

**Table 2:** Comparison of prediction error between EEMD-RNN model and HS-EEMD-RNN mode.

Models	MAE	RMSE	MAPE
EEMD-RNN	0.221	0.250	0.123
HS-EEMD-RNN	0.088	0.101	0.048

**Table 3:** Comparison of predicted values.

Samples	The predicted value affects the ratio		RMSE	
	HS-EEMD-RNN	EEMD-RNN	HS-EEMD-RNN	EEMD-RNN
1	0.4	0.2	0.34	4.10
2	0.7	0.6	8.20	23.82
3	0.6	0.4	1.87	6.22
4	0.6	0.5	3.76	8.17
5	0.6	0.4	1.12	15.36
6	0.6	0.3	3.63	8.79
7	0.4	0.2	16.71	42.22
Ava	—	—	8.91	27.17

## Data Availability

The dataset can be accessed upon request.
